The article "Agreement of total corneal power between 2 swept-source optical coherence tomography and Scheimpflug tomography in normal and keratoconic patients" was published in 2022. Journal: PLoS One.

# Agreement of total corneal power between 2 swept-source optical coherence tomography and Scheimpflug tomography in normal and keratoconic patients

**DOI:** 10.1371/journal.pone.0268856

**Published:** 2022-05-24

**Authors:** Rosepon Asawaworarit, Vannarut Satitpitakul, Parichart Taweekitikul, Krit Pongpirul

**Affiliations:** 1 Department of Ophthalmology, Faculty of Medicine, Excellence Center for Cornea and Limbal Stem Cell Transplantation, King Chulalongkorn Memorial Hospital, Chulalongkorn University, Bangkok, Thailand; 2 Faculty of Medicine, Chulalongkorn University, Bangkok, Thailand; University of Missouri-Columbia, UNITED STATES

## Abstract

**Purpose:**

To evaluate agreement of total corneal power (TCP) measured by swept-source anterior segment optical coherence tomography (CASIA 2), Scheimpflug tomography (Pentacam AXL), and swept-source optical biometer (IOLMaster 700) in normal and keratoconic patients.

**Methods:**

This is a prospective observational study conducted at King Chulalongkorn Memorial Hospital, Bangkok, Thailand. Biometric values were measured by each device for three times by two operators to evaluate repeatability and reproducibility of TCP. The agreement of TCP and other parameters including total corneal astigmatism, anterior keratometry, anterior corneal astigmatism, posterior keratometry, posterior corneal astigmatism, anterior chamber depth, white-to-white corneal diameter (WTW), central corneal thickness, and intraocular power were also evaluated.

**Results:**

This study enrolled 100 healthy participants and 34 patients with keratoconus. The repeatability and reproducibility of TCP were high in all devices (ICC > 0.9). The agreement of TCP was excellent among three devices in both groups (ICC > 0.9). However, the agreement of TCP between CASIA 2 and IOLMaster 700 was slightly lower in healthy participants (ICC = 0.867) and keratoconic patients (ICC = 0.852) with mean differences of more than 1.0 diopter is clinically significant. Wider 95% limit of agreement were found in keratoconic eyes. Most of other parameters showed good to excellent agreement except WTW which showed poor to moderate agreement in both groups. IOL power showed clinically significant differences in patients with keratoconus.

**Conclusions:**

The agreement of TCP measured by three devices was excellent in normal and keratoconic patients. However, TCP cannot be used interchangeably between devices.

## Introduction

One of the keys to achieving a favorable refractive outcome after cataract surgery is the precise ocular biometer values. Ocular biometric values are generally used for intraocular lens (IOL) power calculation and surgical planning, such as incision wound location and length of incisional correction. IOL calculation and surgical planning have mainly relied on keratometry value of the anterior corneal surface and the standardized keratometric index of refraction (1.3375) [1]. Recent studies have demonstrated that assessment of posterior corneal curvature provides benefits in patients’ refractive outcome [2]. Moreover, the variability of posterior corneal curvature in normal and especially in keratoconic eyes can lead to a significant difference between the measurement of anterior corneal surface alone with refractive index to simulate the total refractive power of cornea, and the direct measurement of total corneal power (TCP) [3, 4].

In recent years, several biometric devices directly measuring TCP based on different principles have been developed. IOLMaster 700 (Carl Zeiss Meditec AG, Jena, Germany), a swept-source optical coherence tomography (SS-OCT), is one of the most widely used optical biometers for IOL power calculation. IOLMaster 700 allows the assessment of posterior corneal curvature by incorporating the anterior corneal data taken by telecentric keratometry with corneal thickness taken by SS-OCT [5]. Pentacam AXL (Oculus Optikgerate GmbH, Wetzlar, Germany) uses a single rotating Scheimpflug camera combined with partial coherence interferometry to directly measure both anterior and posterior corneal surface as well as the other ocular biometry. CASIA 2 (Tomey Corp., Nagoya, Japan), a latterly introduced anterior segment optical coherence tomography is an SS-OCT-based device which is specifically designed and used for cross-sectional imaging of the anterior segment structure of the eye with high resolution and high scan speed, allowing the anterior and posterior corneal curvature to be obtained. In addition, both Pentacam AXL and CASIA 2 also provide additional IOL calculation features as well.

The purpose of this study was to evaluate the repeatability and reproducibility of TCP and the agreement of TCP and other biometric parameters including total corneal astigmatism (TCA), anterior keratometry (anterior K), anterior corneal astigmatism (ACA), posterior keratometry (posterior K), posterior corneal astigmatism (PCA), anterior chamber depth (ACD), white-to-white (WTW), central corneal thickness (CCT), and IOL powers obtained from CASIA 2, Pentacam AXL and IOLMaster 700 in normal and keratoconic patients.

## Materials and methods

This prospective cross-sectional study included 100 normal eyes of 100 participants and 34 eyes of 34 participants with either subclinical keratoconus or keratoconus stage 1–3 according to Amsler-Krumeich classification [6]. The study was performed following the tenets of the Declaration of Helsinki and was approved by the Institutional Review Board, Faculty of Medicine, Chulalongkorn University, Bangkok, Thailand. Written informed consents were obtained from all participants.

Exclusion criteria were a history of corneal trauma or surgery, any ocular diseases other than cataracts and history of corneal hydrops. The patient’s right eye was included in this study unless it met the exclusion criteria. In such case, the left eye would be enrolled instead.

Participants’ biometric values were measured by three devices including CASIA 2, Pentacam AXL and IOLMaster 700. The order of measurement by these 3 devices was randomly assigned since the sequence of the measurement may affect on the biometric values from each device due to the changes in participants’ ocular surface and attention. All devices were calibrated each day before the first measurement following the manufacturers’ instructions. A standard methodology to take measurements on each device was used. During measurement, all participants were instructed to keep their chin and forehead in position and look at the fixation light. Complete blinking was required before each automatic capture. After finishing each measurement, a short break was allowed. The device was realigned to the default position before subsequent measurement. The measurement was accepted for analysis if image quality status “OK” showed on the device screen. Otherwise, the measurement would be repeated until a good-quality image was acquired.

For each device, the first experienced operator performed two consecutive measurements for an intra-observer repeatability assessment. The second experienced operator then performed one measurement for an inter-observer reproducibility assessment.

The measured parameters, including TCP, TCA (vector summation of anterior and posterior corneal astigmatism), anterior K, ACA, posterior K, PCA, ACD, WTW and CCT were recorded. Vector analysis for astigmatism was also evaluated in J(0) and J(45) [7].

IOL powers were then calculated from each device using SRK/T and Barrett Universal II formulas. Anterior K with standardized keratometric index of refraction (1.3375) was used to calculate IOL powers in both normal and keratoconic eyes. Because CASIA 2 cannot measure the axial length, the axial length obtained from IOLMaster 700 was used to calculate IOL power. Acrysof SN60WF (Alcon Laboratories, Fort Worth, Texas, USA) was used as a model for IOL calculation.

### Statistical analysis

TCP was used to evaluate the repeatability and reproducibility of each device. The repeatability or intra-observer reliability was analyzed using the two measurements from the first operator. The reproducibility or inter-observer reliability was analyzed using the first measurement from the first operator and the measurement from the second operator.

The agreement among three devices and the agreement between CASIA 2 and Pentacam AXL, CASIA 2 and IOLMaster 700, and Pentcam AXL and IOLMaster 700 were analyzed using the first measurement of each device.

Intraclass correlation coefficient (ICC) and Bland-Altman plot with 95% limits of agreement (LoA) [8] were used to evaluate the repeatability, reproducibility, and the agreement between devices. Within-subject SD (Sw), test-retest repeatability, and within-subject coefficient of variation (CoV) were also used to evaluate the repeatability and reproducibility. Within-subject SD was calculated as the square of mean of within-subject variance. Test-retest repeatability was defined as Sw multiply by √2 × 1.96 (= 2.77). This value indicates that the interval between measurements for the same subject is expected to be less than Sw x 2.77 for 95% of pairs of measurement [9]. CoV was calculated by ratio of within-subject SD to mean [10]. Low values of within-subject SD, test-retest repeatability and CoV were considered better repeatability. ICC was classified as follows: ICC of less than 0.5 was considered poor agreement; ICC of 0.5 to less than 0.75 was considered moderate agreement; ICC of 0.75 to less than 0.90 was considered good agreement; and, ICC of 0.90 or more was considered excellent agreement [11]. *P* value < 0.05 was considered statistically significant. Statistical analysis was performed using SPSS software (version 23.0, SPSS, Inc.).

## Results and discussion

One hundred and thirty-four participants (100 normal and 34 keratoconic eyes) completed all measurements and were eligible for analysis. Mean age of the entire participants was 34.86 ±13.34 years (range 18 to 71 years). Demographic data of the study population is shown in Table 1.

**Table 1:** Demographic data.

Demographic data	Normal	Keratoconus	*P* value^a^
	(n = 100)	(n = 34)	
Age, mean ± SD (range, years)	36.72 ± 14.26 (18–71)	29.38 ± 8.10 (19–57)	<0.01
Sex, female, n (%)	84 (84%)	13 (38.24%)	<0.01
Right eye, n (%)	92 (92%)	21 (61.76%)	<0.01
Uncorrected distance visual acuity, mean ± SD (LogMAR)	0.63 ± 0.58	0.75 ± 0.52	0.31
Manifest spherical equivalent, mean ± SD (diopters)	-3.57 ± 3.95	-6.11 ± 3.70	<0.01
Sphere	-3.21 ± 3.83	-4.27 ± 3.33	0.15
Cylinder	-0.67 ± 0.56	-3.60 ± 2.38	<0.01
Amsler—Krumeich keratoconus stage, n (%)			
Stage 1		25 (73.53%)	
Stage 2		6 (17.65%)	
Stage 3		3 (8.82%)	

^a^ *P* values calculated using independent t test and Chi-square test.

Tables 2 and 3 respectively show the mean biometric parameters obtained from the three devices in normal and keratoconic eyes. Among the three devices, TCP, TCA, J(0) vector of TCA, posterior K, WTW and CCT were significantly different in normal eyes. In keratoconic eyes, TCP and PCA were significantly different.

**Table 2:** Biometric measurements with CASIA 2, Pentacam AXL, and IOLMaster 700 in normal participants.

Parameters	CASIA 2		Pentacam AXL		IOLMaster 700		*P* value			
	Mean ± SD	Range	Mean ± SD	Range	Mean ± SD	Range	3 devices^a^	1 vs 2^b^	1 vs 3^b^	2 vs 3^b^
TCP (D)	43.09 ± 1.31	38.90, 46.10	43.49 ± 1.41	39.50, 47.00	44.11 ± 1.35	40.04, 47.35	<0.01	<0.01	<0.01	<0.01
TCA (D)										
Power (D)	-1.03 ± 0.62	-4.00, -0.20	-1.13 ± 0.69	-4.00, -0.10	-1.10 ± 0.59	-3.02, -0.14	<0.01	0.01	<0.01	<0.01
J(0)	0.41 ± 0.37	-0.45, 1.66	0.46 ± 0.42	-0.58, 1.85	0.43 ± 0.38	-0.52, 1.49	<0.01	0.03	<0.01	<0.01
J(45)	-0.10 ± 0.22	-0.56, 1.12	-0.08 ± 0.22	-0.58, 0.75	-0.09 ± 0.22	-0.63, 0.57	0.35	0.97	0.46	1
Anterior K (D)	44.15 ± 1.33	39.80, 47.10	44.05 ± 1.32	40.00, 47.30	44.13 ± 1.35	39.97, 47.36	0.86	1	1	1
ACA										
Power (D)	-1.17 ± 0.66	-4.30, -0.20	-1.18 ± 0.77	-3.60, 2.50	-1.15 ± 0.59	-2.94, -0.18	0.94	1	1	1
J(0)	0.50 ± 0.37	-0.39, 1.82	0.51 ± 0.42	-1.23, 1.67	0.48 ± 0.37	-0.49, 1.45	0.77	1	1	1
J(45)	-0.10 ± 0.23	-0.57, 1.14	-0.08 ± 0.21	-0.59, 0.67	-0.08 ± 0.21	-0.68, 0.58	0.86	1	1	1
Posterior K (D)	-6.24 ± 0.20	-6.80, -5,50	-6.38 ± 0.21	-7.00, -5.70	-5.95 ± 0.19	-6.46, -5.30	<0.01	0.07	<0.01	<0.01
PCA										
Power (D)	-0.32 ± 0.12	-0.80, -0.10	-0.37 ± 0.14	-0.80, -0.10	-0.24 ± 0.11	-0.50, 0.00	0.55	0.86	1	1
J(0)	47.89 ± 0.06	-0.35, 0.01	-0.18 ± 0.07	-0.39, -0.01	-0.11 ± 0.06	-0.25, 0.05	0.67	1	1	1
J(45)	0.02 ± 0.04	-0.19, 0.11	0.01 ± 0.05	-0.10, 0.16	0.01 ± 0.05	-0.10, 0.16	0.84	1	1	1
ACD (mm)	3.53 ± 0.39	2.52. 4.24	3.46 ± 0.39	2.46, 4.18	3.43 ± 0.39	2.41, 4.14	0.18	0.75	0.21	1
WTW (mm)	11.76 ± 0.51	9.14, 12.64	11.71 ± 0.42	10.8, 13.5	11.91 ± 0.59	8.40, 12.80	0.02	1	0.16	0.02
CCT (μm)	528.21 ± 28.67	446, 621	539.55 ± 28.06	458, 632	534.1 ± 30.74	447, 627	0.02	0.02	0.46	0.56
IOL power (D)										
SRK/T	16.91 ± 5.17	5.0, 25.5	17.02 ± 5.08	5.0, 25.0	16.93 ± 5.17	4.5, 25.5	0.99	1	1	1
Barrett Universal II	16.91 ± 5.17	6.0, 25.5	17.01 ± 5.12	5.5, 25.5	16.83 ± 5.15	5.5, 25.5	0.97	1	1	1

TCP = total corneal power; TCA = total corneal astigmatism; Anterior K = anterior keratometry; ACA = anterior corneal astigmatism; Posterior K = posterior keratometry; PCA = posterior corneal astigmatism; ACD = anterior chamber depth; WTW = white-to-white; CCT = central corneal thickness; IOL = intraocular lens; J(0) = Jackson cross-cylinder, axes at 0 degrees and 90 degrees; J(45) = Jackson cross-cylinder, axes at 45 degrees and 135 degrees; D = diopters

^a^ *P* values calculated using ANOVA test.

^b^ *P* values calculated using Bonferroni multiple-comparison test.

**Table 3:** Biometric measurements with CASIA 2, Pentacam AXL, and IOLMaster 700 in keratoconic participants.

Parameters	CASIA 2		Pentacam AXL		IOLMaster 700		*P* value			
	Mean ± SD	Range	Mean ± SD	Range	Mean ± SD	Range	3 devices^a^	1 vs 2^b^	1 vs 3^b^	2 vs 3^b^
TCP (D)	45.39 ± 2.47	40.40, 52.40	45.98 ± 2.9	40.90, 53.20	47.27 ± 3.75	41.58, 56.33	0.01	0.67	0.20	<0.01
TCA (D)										
Power (D)	-3.22 ± 1.74	-7.50, -0.80	-3.75 ± 2.14	-10.30, -0.90	-4.66 ± 2.79	-11.00, -0.25	0.64	1	1	1
J(0)	1.30 ± 1.09	-1.29, 3.74	1.55 ± 1.30	-0.71, 5.10	1.40 ± 2.04	-3.42, 5.47	0.25	1	0.44	0.45
J(45)	-0.28 ± 0.66	-1.57, 1.58	-0.01 ± 0.79	-1.82, 1.72	-0.12 ± 1.17	-2.72, 2.59	0.25	0.64	0.35	1
Anterior K (D)	46.66 ± 2.65	41.60, 53.90	47.08 ± 3.33	41.60, 54.60	47.39 ± 3.85	41.67, 56.49	0.66	1	1	1
ACA										
Power (D)	-3.47 ± 1.82	-7.80, -0.80	-3.95 ± 2.29	-11.5, -0.7	-4.73 ± 2.81	-12.00, -0.32	0.09	1	0.09	0.51
J(0)	1.44 ± 1.09	-1.00, 3.90	1.44 ± 1.54	-1.94, 5.62	1.44 ± 2.06	-3.30, 5.97	1	1	1	1
J(45)	-0.33 ± 0.69	-1.62, 1.64	-0.03 ± 0.92	-1.93, 1.58	-0.12 ± 1.17	-2.77, 2.60	0.40	0.57	1	1
Posterior K (D)	-6.77 ± 0.53	-7.90, -6.00	-6.95 ± 0.67	-8.30, -5.90	-6.49 ± 0.64	-7.85, -5.59	0.04	1	0.04	0.26
PCA										
Power (D)	-0.72 ± 0.29	-1.40, -0.10	-0.79 ± 0.47	-2.20, 0.00	-0.71 ± 0.39	-1.79, -0.11	0.03	1	0.03	0.30
J(0)	-0.32 ± 0.16	-0.67, 0.04	-0.32 ± 0.28	-1.09, 0.17	-0.23 ± 0.28	-0.89, 0.34	0.79	1	1	1
J(45)	0.09 ± 0.13 df	-0.22, 0.34	0.04 ± 0.19	-0.43, 0.45	0.03 ± 0.19	-0.37, 0.44	0.46	0.64	1	1
ACD (mm)	3.79 ± 0.28	3.12, 4.18	3.73 ± 0.29	3.11, 4.21	3.69 ± 0.28	3.01, 4.08	0.37	1	0.49	1
WTW (mm)	11.87 ± 0.49	10.93, 12.68	11.83 ± 0.38	11.20, 12.70	12.03 ± 0.71	8.80, 12.90	0.28	1	0.65	0.41
CCT (μm)	488.79 ± 31.13	414, 565	493.32 ± 31.88	422, 571	493.09 ± 33.33	416, 574	0.81	1	1	1
IOL power (D)										
SRK/T	13.84 ± 4.28	1.5, 21.5	12.88 ± 5.73	-5.5, 21.5	12.31 ± 6.71	-10.0, 21.5	0.53	1	0.80	1
Barrett Universal II	13.37 ± 4.35	3. 21.5	12.65 ± 3.02	-2.0, 21.5	12.06 ± 5.97	-5.5, 21.5	0.59	1	0.91	1

TCP = total corneal power; TCA = total corneal astigmatism; Anterior K = anterior keratometry; ACA = anterior corneal astigmatism; Posterior K = posterior keratometry; PCA = posterior corneal astigmatism; ACD = anterior chamber depth; WTW = white-to-white; CCT = central corneal thickness; IOL = intraocular lens; J(0) = Jackson cross-cylinder, axes at 0 degrees and 90 degrees; J(45) = Jackson cross-cylinder, axes at 45 degrees and 135 degrees; D = diopters

^a^ *P* values calculated using ANOVA test.

^b^ *P* values calculated using Bonferroni multiple-comparison test.

### Repeatability and reproducibility

Within-subject SD, test-retest repeatability, CoV, and ICC of TCP measured by the three devices in normal and keratoconic eyes are demonstrated in Table 4. Both repeatability and reproducibility of all devices are high. The ICCs for the repeatability ranged from 0.996 to 0.997 in normal eyes, and 0.998 to 0.999 in keratoconic eyes. All devices showed low mean differences between the measurements by the same operator, narrow 95% confidence limits (CL) of the ICCs and 95% limits of agreement (LoAs) in both groups of participants. The repeatability of IOLMaster 700 had a much higher mean difference than CASIA 2 and Pentacam AXL in normal eyes. Keratoconic eyes had higher mean differences between measurements by the same operator compared with normal eyes in all devices.

**Table 4:** Repeatability and reproducibility of total corneal power in normal and keratoconus participants.

Parameters	ICC	95% CL		Difference* (Mean ± SD)	95% LoA		Within- subject SD (Sw)	Test-retest repeatability (2.77 Sw)	Within-subject CoV
		Lower	Upper		Lower	Upper			
**Total corneal power (D)**									
**Normal (n = 100)**									
**Repeatability**									
CASIA 2	0.996	0.994	0.997	-0.007 ± 0.171	-0.342	0.328	0.076	0.211	0.002
Pentacam AXL	0.996	0.994	0.997	-0.006 ± 0.175	-0.349	0.337	0.068	0.188	0.002
IOLMaster 700	0.997	0.995	0.998	0.025 ± 0.152	-0.273	0.323	0.081	0.224	0.002
**Reproducibility**									
CASIA 2	0.998	0.997	0.998	0.000 ± 0.124	-0.243	0.243	0.062	0.172	0.001
Pentacam AXL	0.996	0.995	0.998	-0.003 ± 0.162	0.321	0.315	0.074	0.205	0.002
IOLMaster 700	0.995	0.992	0.997	0.056 ± 0.180	-0.297	0.409	0.095	0.263	0.002
**Keratoconus (n = 34)**									
**Repeatability**									
CASIA 2	0.998	0.997	0.999	-0.038 ± 0.202	-0.434	0.358	0.102	0.283	0.002
Pentacam AXL	0.999	0.997	0.999	-0.059 ± 0.205	-0.461	0.343	0.096	0.266	0.002
IOLMaster 700	0.998	0.997	0.999	0.042 ± 0.312	-0.57	0.654	0.140	0.388	0.003
**Reproducibility**									
CASIA 2	0.996	0.991	0.998	0.012 ± 0.330	-0.635	0.659	0.154	0.427	0.003
Pentacam AXL	0.997	0.995	0.999	-0.103 ± 0.274	-0.64	0.434	0.123	0.341	0.003
IOLMaster 700	0.998	0.997	0.999	0.052 ± 0.298	-0.532	0.636	0.150	0.416	0.003

ICC = intraclass correlation coefficient; D = diopters; CL = confidence limits; LoA = limits of agreement; CoV = coefficient of variation

*Between 2 measurements by the same operator for repeatability analysis and by the different operators for reproducibility analysis.

The ICCs for reproducibility ranged from 0.995 to 0.998 in normal eyes, and 0.996 to 0.998 in keratoconic eyes. All devices showed low mean differences between the measurements by the different operators, and narrow 95% CL of the ICCs and 95% LoAs in both groups of participants. Similar to the repeatability analysis, the reproducibility of IOLMaster 700 had a much higher mean difference than the other devices. Using CASIA 2 and Pentacam AXL, keratoconic eyes had higher mean differences between TCP measured by the different operators compared with normal eyes, while IOLMaster 700 demonstrated comparable mean differences. Among 3 devices, CASIA 2 demonstrated the lowest mean difference in the repeatability and reproducibility analysis in both normal and keratoconic eyes.

### Agreement between the devices

Agreement of TCP among the three devices was excellent in both normal (ICC = 0.996) and keratoconic (ICC = 0.970) eyes. The CL of the ICCs were narrow. Other biometric parameters and IOL power, except for the J(45) vector of PCA and WTW, showed good to excellent agreement (Table 5).

**Table 5:** Agreement among CASIA 2, Pentacam AXL, IOLMaster 700 in normal and keratoconus participants.

Parameters	Normal (n = 100)			Keratoconus (n = 34)		
	ICC	95% CL		ICC	95% CL	
		Lower	Upper		Lower	Upper
TCP (D)	0.996	0.994	0.997	0.970	0.948	0.984
TCA (D)						
Power (D)	0.893	0.850	0.925	0.901	0.825	0.947
J(0)	0.938	0.913	0.956	0.926	0.869	0.960
J(45)	0.812	0.738	0.868	0.884	0.795	0.938
Anterior K (D)	0.996	0.995	0.997	0.980	0.964	0.989
ACA						
Power (D)	0.878	0.830	0.914	0.934	0.883	0.965
J(0)	0.919	0.887	0.943	0.945	0.902	0.971
J(45)	0.830	0.763	0.881	0.922	0.863	0.959
Posterior K (D)	0.982	0.975	0.988	0.990	0.982	0.995
PCA						
Power (D)	0.882	0.835	0.917	0.915	0.851	0.955
J(0)	0.903	0.865	0.932	0.903	0.828	0.948
J(45)	0.452	0.236	0.615	0.600	0.294	0.787
ACD (mm)	0.999	0.999	1.000	0.997	0.995	0.999
WTW (mm)	0.547	0.368	0.682	0.670	0.418	0.824
CCT (μm)	0.995	0.993	0.997	0.993	0.987	0.996
IOL power (D)						
SRK/T	0.999	0.999	1.000	0.971	0.948	0.984
Barrett Universal II	0.999	0.999	0.999	0.983	0.970	0.991

TCP = total corneal power; TCA = total corneal astigmatism; Anterior K = anterior keratometry; ACA = anterior corneal astigmatism; Posterior K = posterior keratometry; PCA = posterior corneal astigmatism; ACD = anterior chamber depth; WTW = white-to-white; CCT = central corneal thickness; IOL = intraocular lens; J(0) = Jackson cross-cylinder, axes at 0 degrees and 90 degrees; J(45) = Jackson cross-cylinder, axes at 45 degrees and 135 degrees; D = diopters; ICC = intraclass correlation coefficient; CL = confidence limits.

Comparison between any two devices is shown in Tables 6 and 7. The agreement of TCP between Pentacam AXL and the other devices was excellent (ICCs ranged from 0.931 to 0.966), and between CASIA 2 and IOLMaster 700 was good (ICCs ranged from 0.851 to 0.867) in both groups of participants. The mean differences between TCP from Pentacam AXL and the other devices in normal eyes and Pentacam AXL and CASIA 2 in keratoconic eyes were less than 1 diopter, while the other comparisons were more than 1 diopter. The 95% LoAs between the TCP from any two devices were narrow in normal eyes, but the 95% LoAs were much wider in keratoconic eyes. The Bland-Altman plot of TCP showed that the mean differences between any two devices increased with the mean TCP in keratoconic eyes (Fig 1).

**Fig 1:** Bland-Altman plots of total corneal power between devices in normal and keratoconic eyes. Bland-Altman plots showing the agreement of total corneal power between CASIA 2 and Pentacam AXL (A, D), CASIA 2 and IOLMaster 700 (B, E) and Pentacam AXL and IOLMaster 700 (C, F) in healthy (A-C) and keratoconic (D-F) participants. The middle-dashed line shows the mean difference, and the top and bottom dashed lines show the upper and lower 95% limits of agreement, respectively.

**Table 6:** Agreement between CASIA 2 and Pentacam AXL, CASIA 2 and IOLMaster 700, and Pentacam AXL and IOLMaster 700 in normal eyes.

Parameters	CASIA 2 and Pentacam AXL						CASIA 2 and IOLMaster 700						Pentacam AXL and IOLMaster 700					
	ICC	95% CL		Difference)	95% LoA		ICC	95% CL		Difference	95% LoA		ICC	95% CL		Difference	95% LoA	
		Lower	Upper	(Mean ± SD)	Lower	Lower		Upper	Lower	(Mean ± SD)	Upper	Lower		Upper	Lower	(Mean ± SD)	Upper	Lower
TCP (D)	0.966	0.180	0.991	-0.432 ± 0.242	-0.906	0.042	0.867	-0.019	0.970	-1.025 ± 0.177	-1.372	-0.679	0.947	-0.038	0.988	-0.593 ± 0.224	-1.032	-0.155
TCA (D)																		
Power (D)	0.852	0.779	0.901	0.096 ± 0.467	-0.818	1.011	0.867	0.802	0.910	0.065 ± 0.412	-0.743	0.873	0.819	0.731	0.878	-0.031 ± 0.505	-1.020	0.958
J0	0.909	0.864	0.939	-0.049 ± 0.224	-0.488	0.389	0.929	0.894	0.952	-0.023 ± 0.193	-0.401	0.355	0.889	0.836	0.925	0.026 ± 0.252	-0.467	0.520
J45	0.793	0.692	0.860	-0.018 ± 0.182	-0.374	0.338	0.639	0.462	0.757	-0.006 ± 0.226	-0.448	0.436	0.788	0.685	0.857	0.012 ± 0.181	-0.344	0.367
Anterior K (D)	0.992	0.984	0.996	0.102 ± 0.208	-0.306	0.510	0.996	0.994	0.997	0.028 ± 0.172	-0.309	0.364	0.993	0.988	0.996	-0.074 ± 0.213	-0.492	0.343
ACA																		
Power (D)	0.834	0.754	0.889	0.011 ± 0.540	-1.048	1.069	0.866	0.801	0.910	-0.022 ± 0.429	-0.862	0.818	0.790	0.688	0.859	-0.033 ± 0.570	-1.149	1.084
J0	0.880	0.821	0.919	-0.013 ± 0.261	-0.524	0.499	0.923	0.886	0.948	0.027 ± 0.196	-0.358	0.411	0.849	0.776	0.899	0.039 ± 0.286	-0.522	0.600
J45	0.820	0.732	0.878	-0.017 ± 0.173	-0.355	0.322	0.680	0.525	0.785	-0.012 ± 0.218	-0.439	0.414	0.791	0.690	0.860	0.004 ± 0.178	-0.345	0.354
Posterior K (D)	0.843	-0.141	0.956	0.141 ± 0.062	0.019	0.263	0.638	-0.037	0.898	-0.287 ± 0.058	-0.401	-0.172	0.422	-0.039	0.784	-0.428 ± 0.074	-0.573	-0.283
PCA																		
Power (D)	0.851	0.655	0.923	0.049 ± 0.080	-0.107	0.205	0.684	0.134	0.853	-0.084 ± 0.095	-0.269	0.102	0.602	-0.195	0.840	-0.133 ± 0.100	-0.328	0.063
J0	0.860	0.686	0.926	0.024 ± 0.040	-0.055	0.102	0.721	-0.024	0.89	-0.047 ± 0.043	-0.131	0.037	0.630	-0.211	0.862	-0.071 ± 0.049	-0.166	0.024
J45	0.823	0.737	0.881	0.007 ± 0.036	-0.064	0.077	0.707	0.565	0.803	0.009 ± 0.043	-0.074	0.093	0.689	0.537	0.791	0.003 ± 0.046	-0.088	0.094
ACD (mm)	0.992	0.318	0.998	0.064 ± 0.024	0.017	0.110	0.982	0.055	0.996	0.101 ± 0.025	0.053	0.149	0.997	0.907	0.999	0.037 ± 0.026	-0.014	0.088
WTW (mm)	0.525	0.263	0.695	0.062 ± 0.533	-0.984	1.107	0.338	-0.005	0.566	-0.147 ± 0.707	-1.532	1.238	0.492	0.241	0.661	-0.204 ± 0.594	-1.369	0.961
CCT (μm)	0.956	-0.020	0.990	-11.340 ± 4.262	-19.694	-2.986	0.986	0.633	0.996	-5.890 ± 3.923	-13.579	1.799	0.980	0.894	0.992	5.450 ± 6.315	-6.928	17.828
IOL power (D)																		
SRK/T	0.999	0.998	0.999	-0.110 ± 0.345	-0.786	0.566	0.999	0.999	1.000	-0.015 ± 0.261	-0.526	0.496	0.999	0.998	0.999	0.095 ± 0.324	-0.539	0.729
BU-II	0.999	0.998	0.999	-0.095 ± 0.374	-0.828	0.638	0.999	0.998	0.999	0.085 ± 0.326	-0.554	0.724	0.998	0.997	0.999	0.180 ± 0.373	-0.551	0.911

TCP = total corneal power; TCA = total corneal astigmatism; Anterior K = anterior keratometry; ACA = anterior corneal astigmatism; Posterior K = posterior keratometry; PCA = posterior corneal astigmatism; ACD = anterior chamber depth; WTW = white-to-white; CCT = central corneal thickness; IOL = intraocular lens; J0 = Jackson cross-cylinder, axes at 0 degrees and 90 degrees; J45 = Jackson cross-cylinder, axes at 45 degrees and 135 degrees; BU-II = Barrett Universal II; D = diopters; ICC = intraclass correlation coefficient; CL = confidence limits; LoA = limits of agreement.

**Table 7:** Agreement between CASIA 2 and Pentacam AXL, CASIA 2 and IOLMaster 700, and Pentacam AXL and IOLMaster 700 in keratoconic eyes.

Parameters	CASIA 2 and Pentacam AXL						CASIA 2 and IOLMaster 700						Pentacam AXL and IOLMaster 700					
	ICC	95% CL		Difference)	95% LoA		ICC	95% CL		Difference	95% LoA		ICC	95% CL		Difference	95% LoA	
		Lower	Upper	(Mean ± SD)	Lower	Lower		Upper	Lower	(Mean ± SD)	Upper	Lower		Upper	Lower	(Mean ± SD)	Upper	Lower
TCP (D)	0.966	0.864	0.987	-0.591 ± 0.806	-2.171	0.988	0.851	0.107	0.953	-1.881 ± 1.633	-5.082	1.321	0.931	0.486	0.979	-1.289 ± 1.218	-3.676	1.097
TCA (D)																		
Power (D)	0.914	0.786	0.961	0.529 ± 0.998	-1.427	2.486	0.743	0.240	0.894	1.439 ± 1.809	-2.106	4.985	0.813	0.585	0.911	0.910 ± 1.841	-2.698	4.518
J0	0.953	0.875	0.979	-0.251 ± 0.457	-1.147	0.645	0.851	0.702	0.926	-0.099 ± 1.188	-2.426	2.229	0.896	0.793	0.948	0.152 ± 1.054	-1.915	2.218
J45	0.855	0.629	0.935	-0.272 ± 0.466	-1.185	0.640	0.855	0.712	0.927	-0.156 ± 0.669	-1.467	1.155	0.787	0.575	0.893	0.116 ± 0.836	-1.523	1.755
Anterior K (D)	0.970	0.931	0.986	-0.426 ± 0.953	-2.295	1.442	0.934	0.844	0.969	-0.734 ± 1.516	-3.705	2.237	0.986	0.970	0.993	-0.307 ± 0.791	-1.857	1.242
ACA																		
Power (D)	0.928	0.830	0.967	0.479 ± 0.989	-1.458	2.417	0.767	0.372	0.899	1.263 ± 1.817	-2.299	4.824	0.919	0.755	0.966	0.783 ± 1.224	-1.616	3.183
J0	0.948	0.896	0.974	0.005 ± 0.599	-1.170	1.179	0.848	0.695	0.924	0.005 ± 1.209	-2.365	2.374	0.961	0.922	0.981	0 ± 0.714	-1.399	1.399
J45	0.863	0.639	0.940	-0.303 ± 0.504	-1.291	0.684	0.850	0.699	0.925	-0.213 ± 0.676	-1.537	1.112	0.908	0.816	0.954	0.091 ± 0.615	-1.114	1.295
Posterior K (D)	0.957	0.653	0.987	0.182 ± 0.177	-0.164	0.529	0.931	-0.025	0.984	-0.276 ± 0.152	-0.573	0.021	0.883	-0.044	0.975	-0.459 ± 0.115	-0.684	-0.234
PCA																		
Power (D)	0.828	0.658	0.913	0.074 ± 0.296	-0.506	0.653	0.846	0.691	0.923	-0.008 ± 0.253	-0.504	0.488	0.927	0.845	0.964	-0.082 ± 0.215	-0.503	0.339
J0	0.860	0.719	0.930	-0.001 ± 0.159	-0.313	0.311	0.794	0.547	0.902	-0.086 ± 0.175	-0.429	0.256	0.950	0.686	0.983	-0.086 ± 0.091	-0.265	0.093
J45	0.781	0.553	0.892	0.052 ± 0.132	-0.207	0.310	0.777	0.508	0.894	0.065 ± 0.128	-0.186	0.316	0.942	0.885	0.971	0.013 ± 0.088	-0.159	0.185
ACD (mm)	0.986	0.729	0.996	0.054 ± 0.042	-0.027	0.136	0.968	0.006	0.994	0.096 ± 0.032	0.034	0.158	0.991	0.846	0.998	0.041 ± 0.033	-0.023	0.106
WTW (mm)	0.713	0.407	0.861	0.009 ± 0.415	-0.804	0.823	0.512	0.035	0.756	-0.175 ± 0.695	-1.537	1.188	0.559	0.135	0.779	-0.197 ± 0.625	-1.422	1.028
CCT (μm)	0.983	0.942	0.993	-4.529 ± 6.890	-18.033	8.974	0.987	0.948	0.995	-4.294 ± 5.865	-15.789	7.201	0.988	0.976	0.994	0.235 ± 7.237	-13.948	14.419
IOL power (D)																		
SRK/T	0.955	0.891	0.980	0.956 ± 1.904	-2.777	4.688	0.898	0.765	0.952	1.529 ± 3.169	-4.682	7.741	0.983	0.964	0.992	0.574 ± 1.523	-2.412	3.559
BU-II	0.973	0.932	0.988	0.721 ± 1.394	-2.011	3.452	0.939	0.828	0.974	1.309 ± 2.202	-3.007	5.625	0.987	0.966	0.994	0.588 ± 1.171	-1.706	2.883

TCP = total corneal power; TCA = total corneal astigmatism; Anterior K = anterior keratometry; ACA = anterior corneal astigmatism; Posterior K = posterior keratometry; PCA = posterior corneal astigmatism; ACD = anterior chamber depth; WTW = white-to-white; CCT = central corneal thickness; IOL = intraocular lens; J0 = Jackson cross-cylinder, axes at 0 degrees and 90 degrees; J45 = Jackson cross-cylinder, axes at 45 degrees and 135 degrees; BU-II = Barrett Universal II; D = diopters; ICC = intraclass correlation coefficient; CL = confidence limits; LoA = limits of agreement.

For other biometric parameters, most comparisons demonstrated good to excellent agreement, except J(45) vectors of TCA and ACA between CASIA 2 and IOLMaster 700, posterior K and PCA between IOLMaster 700 and the other two devices, and WTW between any two devices in normal eyes. In participants with keratoconus, most comparisons also displayed good to excellent agreement except TCA between CASIA 2 and IOLMaster 700, and WTW between any two devices.

Agreement of IOL powers calculated by SRK/T and Barrett Universal II formulas was excellent (ICCs ranged from 0.955 to 0.999), except between CASIA 2 and IOLMaster 700 in participants with keratoconus, which showed good agreement (ICC = 0.898). Mean differences of calculated IOL powers from any two devices were lower than 0.5 diopters in normal eyes, but higher than 0.5 diopters in keratoconic eyes. This study showed that repeatability and reproducibility of TCP measured by CASIA 2, Pentacam AXL, and IOLMaster 700 are high. Among the three devices, CASIA 2 showed the lowest mean differences in both repeatability and reproducibility analyses. Agreement of TCP among the three devices was excellent in both normal and keratoconic eyes. However, the mean differences and 95% LoAs between any two devices were respectively higher and wider in keratoconic eyes compared with normal eyes. The Bland-Altman plot in keratoconic eyes demonstrated that increase in TCP tended to show higher mean differences in the TCP among the devices.

CASIA 2, Pentacam AXL, and IOLMaster 700 use different technologies to measure TCP and the other ocular biometers. CASIA 2 is an SS-OCT-based device with a wavelength of 1310 nm. It determines TCP, which is called real keratometry, by measuring anterior corneal surface, posterior corneal surface, and pachymetry, using 16 radial B-scans centered on corneal vertex at 2.5 mm and 3.0 mm zones [12]. Pentacam AXL uses a rotating Scheimpflug camera for keratometry, CCT, and ACD measurements. The TCP measured from Pentacam AXL includes total corneal refractive power and true net power. Total corneal refractive power uses a ray-tracing method with snell’s law to calculate refractive power at any point of the cornea, which the manufacturer says may represent actual refractive power [13]. Total corneal refractive power at 3 mm zone was used as TCP in this study. IOLMaster 700 is an SS-OCT based device with a wavelength of 1055 nm. Eighteen points of telecentric keratometry in 3 zones (1.5, 2.5, 3.5 mm) are used in anterior corneal surface measurement, while the SS-OCT system is implemented in the posterior corneal surface, CCT, ACD, and axial length measurements. Total keratometry from IOLMaster 700 determined by calculated anterior corneal surface, posterior corneal surface, and pachymetry combined with thick lens formula [14], was used as TCP in this study.

TCP measured by the three devices had excellent repeatability, reproducibility, and agreement. Our results were similar to previous reports that showed high repeatability of TCP measured by Pentacam AXL [3, 15] and IOLMaster 700 [3, 16]. However, the repeatability and reproducibility of TCP measured by CASIA 2 have not been studied before. Among the three devices, CASIA 2 showed the best repeatability and reproducibility in terms of mean differences in both normal and keratoconic eyes. This might be associated with different principles of ocular biometric measurements and calculations between the devices. Moreover, CASIA 2 required a shorter time to scan an eye when compared with the other devices. The measurement speed of CASIA 2 is 50,000 A-scans per second requiring 0.34 seconds for each measurement, while the scan speed of IOLMaster 700 is 2,000 A-scans per second and the time required for each measurement of Pentacam AXL is 1 second [17]. The shorter time required for measurement contributes to fewer motion artifacts associated with eye movement and patient fatigue.

In this study, we found that TCP obtained from IOLMaster 700 had the highest value, followed by Pentacam AXL and CASIA 2 respectively. The TCP also showed significant differences between any two devices in normal eyes. When analyzing the agreement of TCP between devices in pairs, CASIA 2 and IOLMaster 700 seemed to provide slightly less agreement (ICC 0.876) with mean difference of more than 1.0 diopter, which may be considered clinically significant. Thus, TCP obtained from different devices should not be used interchangeably.

Previous reports have mentioned less repeatability, reproducibility, and errors in keratometric measurements in keratoconic eyes, especially in the advanced stage of the disease. Less repeatability, reproducibility, and inaccurate keratometry were considered to be due to the irregularity of corneal curvature and tear film, as well as stromal scars beneath the breaks in the Bowman layer [17–20]. Although participants with keratoconus in our study were mainly in the early stage of the disease, within-subject SD, test-retest repeatability and CoV of TCP in keratoconic eyes were higher than healthy eyes. In addition, mean differences in TCP and 95% LoA of the repeatability, reproducibility, and the agreement were, respectively, higher and wider in keratoconic eyes compared with healthy eyes. Of the three devices, the mean differences in TCP of the repeatability, reproducibility, and the agreement in keratoconic eyes ranged from 0.038 to 0.059, 0.012 to 0.103, and 0.591 to 1.881 diopters, respectively. Considering the increase in corneal power of more than 1 diopter as a criterion for keratoconus progression [21], the repeatability and reproducibility of all devices are acceptable, however, the same device should be used for following progression from the early stage of keratoconus.

This study found that most of the other biometric parameters including TCA, anterior K, ACA power, posterior K, ACD, CCT, and IOL power calculated by SRK/T and Barrett Universal II formula showed good to excellent agreement among the three devices. In contrast, posterior K and both the power and meridian of PCA obtained from IOLMaster 700 demonstrated poor to moderate agreement with the other two devices. According to previous reports, the amount of PCA power in the normal population was -0.26 to -0.76 diopters [22]. Thus, the mean differences in PCA power ranging from 0.049 to 0.133 diopters in this study seem to be clinically significant. Similarly, with previous reports [3, 16, 19, 23], the agreement in the meridian of TCA, ACA, and PCA between the devices varied from moderate to excellent. Repeated measurements of the astigmatic meridian should be considered. WTW also showed poor to moderate agreement among the three devices. This could be due to the different techniques of WTW measurement in each device. Using Pentacam AXL and IOLMaster 700, WTW is measured automatically from the greyscale step to determine limbus in the photograph. Therefore, any factors, including the darkness, device’s shadow or patients’ nose or lashes, may affect the results [24]. CASIA 2 uses the anterior chamber angle as a landmark and provides angle-to-angle distance [25]. Resembling TCP, the other biometric parameters in keratoconic eyes showed higher mean differences and a wider 95% LoA compared with normal eyes.

Despite some of the optical biometers showing significant differences between the three devices, the IOL powers were similar in normal eyes. The mean differences in IOL power using SRK/T and Barrett Universal II formulas ranged from -0.110 to 0.095 and -0.095 to 0.180 diopters, respectively. With IOLs commercially available in 0.5 diopters increment, the IOL power derived from each device seems to be interchangeable. This might infer that the IOL constants recommended by the manufacturer can be used with no clinically significant difference. In contrast to normal eyes, the mean differences in IOL power in keratoconic eyes were high, which ranged from 0.574 to 1.529 using SRK/T formula and 0.588 to 1.309 using Barrett Universal II formula. In this study, the anterior K was used for IOL power calculation in both normal and keratoconic eyes due to the unavailability of common IOL formula that can be used with TCP. Axial length was not the parameter that was evaluated because CASIA 2 cannot measure it. Instead, axial length from IOLMaster 700 was used for IOL power calculation in CASIA 2. Axial length measurement between IOLMaster 700 and Pentacam AXL showed excellent agreement in many recent studies. IOL power calculation in keratoconus is still challenging for many reasons, including abnormality in anterior and posterior corneal surface, change in corneal refractive index, inaccurate keratometry, alteration of lens’ effective position, and no designed IOL formula available for keratoconic eyes [26, 27].

Our findings are limited to normal eyes without any eye pathology or surgery other than cataract and eyes with early stage keratoconus. A few participants with advanced keratoconus were included in this study. A small number of participants with some degrees of cataract were enrolled.

## Conclusions

The repeatability and reproducibility of TCP obtained from CASIA 2, Pentacam AXL, and IOLMaster 700 are high and comparable in both healthy and keratoconic eyes. TCP and other biometric parameters except for posterior K, PCA, astigmatic meridian, and WTW demonstrated good to excellent agreement among the devices. However, TCP of each device was different and should not be used interchangeably. The discrepancy in TCP and other biometric parameters among the three devices was higher in keratoconic eyes compared with normal eyes.

## Supporting information

S1 Data Minimal anonymized data. (XLSX)
